# A Dual Role for SAGA-Associated Factor 29 (SGF29) in ER Stress Survival by Coordination of Both Histone H3 Acetylation and Histone H3 Lysine-4 Trimethylation

**DOI:** 10.1371/journal.pone.0070035

**Published:** 2013-07-23

**Authors:** Andrea W. Schram, Roy Baas, Pascal W. T. C. Jansen, Anne Riss, Laszlo Tora, Michiel Vermeulen, H. Th. Marc Timmers

**Affiliations:** 1 Department of Molecular Cancer Research, University Medical Center Utrecht, Utrecht, The Netherlands; 2 Cellular Signaling and Nuclear Dynamics Program, Institut de Génétique et de Biologie, Université de Strasbourg, Illkirch, France; George Mason University, United States of America

## Abstract

The SGF29 protein binds to tri-methylated lysine-4 of histone H3 (H3K4me3), which is a histone modification associated with active promoters. Human SGF29 is a subunit of the histone acetyltransferase module of the SAGA (Spt-Ada-Gcn5 acetyltransferase) and ATAC (Ada-Two-A-containing 2A) co-activator complexes. Previous work revealed that the SAGA complex is recruited to endoplasmic reticulum (ER) stress target genes and required for their induction. Here, we report the involvement of SGF29 in the survival of human cells from ER stress. SGF29 knockdown results in impaired transcription of the ER stress genes *GRP78* and *CHOP*. Besides histone H3K14 acetylation, we find that SGF29 is also required for the maintenance of H3K4me3 at these genes, which is already present prior to ER stress. Reduced levels of H3K4me3 in the absence of SGF29 correlate with a decreased association of ASH2L, which is a core component of the SET1/MLL complexes, to *GFP78* and *CHOP*. In conclusion, our results suggest that the H3K4me3-binding protein SGF29 plays a central and dual role in the ER stress response. Prior to ER stress, the protein coordinates H3K4me3 levels, thereby maintaining a ‘poised’ chromatin state on ER stress target gene promoters. Following ER stress induction, SGF29 is required for increased H3K14 acetylation on these genes, which then results in full transcriptional activation, thereby promoting cell survival.

## Background

Eukaryotic transcription is a tightly regulated process, which is controlled by a wide variety of proteins including gene-specific transcription factors, co-regulators and the basal RNA polymerase transcription machinery. Important control mechanisms are exerted at the level of chromatin, of which nucleosomes comprise the basic building block. Post-translational modifications (PTMs) of the histone tails protruding from nucleosomes play a major role in the regulation of transcription and gene expression. The link between PTMs and activation of transcription was stressed by the discovery of the co-activator GCN5 as a histone acetyltransferase (HAT) [1]. Genome-wide localization studies revealed that acetylation of the H3 tail at lysine-9 and -14 (H3K9ac and H3K14ac) are linked with transcriptionally active genes [2–4]. Besides histone acetylation, methylation is also important for gene activity [5–7]. Tri-methylation of lysine-4 on histone H3 (H3K4me3) is strongly associated with the promoters of actively transcribed genes [8–10]. Subsequent studies have shown that both histone acetylations and methylations can serve as recognition sites for chromatin and transcription regulatory complexes. H3K4me3 is recognized by a number of different binding or “reader” domains within proteins such as the Chromo, PHD and double Tudor (Td) domains [11–13]. Well-studied examples of H3K4me3 binders are the PHD finger-containing proteins BPTF, a member of the chromatin remodeling NURF complex [14], and TAF3 [15], a subunit of the basal transcription factor TFIID [16]. TAF3 binds to H3K4me3 with high affinity and can act as a transcriptional co-activator in a PHD finger dependent manner [15,17,18]. Thus, TAF3 forms the molecular link between the active chromatin state of a promoter, and the basal transcription machinery.

Biochemical purifications revealed that in higher eukaryotes GCN5 is part of the evolutionary-conserved SAGA and ATAC co-activator complexes [19,20]. GCN5 is central in their HAT modules, which is consists of the ADA2B, ADA3 and SGF29 proteins in SAGA. ADA2A replaces ADA2B in the HAT module of ATAC [21]. The SAGA complex is composed of ~20 subunits, which are organized into distinct modules. The core of SAGA is formed by SPT20, SPT7, ADA1 and supplemented by several TAF (-like) proteins [22]. Yeast and human SPT20 are highly homologous proteins and they are essential for the structural integrity of the SAGA complex [19,23,24]. Besides the core and HAT modules, SAGA contains modules involved in transcription activation and in de-ubiquitination of histone H2B. Several subunits of SAGA harbor domains capable of interacting with modified chromatin. SPT7 and GCN5 harbor Bromo domains, which can recognize acetylated lysines, and SGF29 contains a double Tudor domain capable of binding H3K4me3 peptides. Indeed, SGF29 is required for binding of the SAGA complex to this mark [25]. Deletion of yeast *SGF29* does not affect SAGA integrity nor composition of the HAT module indicating that SGF29 is a peripheral subunit in this complex [26,27] {Lee, 2011 #214}{Shukla, 2012 #194}. Furthermore, deletion or knockdown of SGF29 leads to decreased global levels of H3K9, K14 and K23 acetylation in yeast and human cells

Yeast SAGA is particularly important for stress-induced transcription [28,29] and this function seems conserved during evolution and extended to both SAGA and ATAC [20]. Genome-localization studies showed that SAGA mostly localizes to gene promoters, whereas ATAC has a preference for gene enhancers [30]. In the human stress response the functions of the SAGA and ATAC complexes also seem to have diverged [20]. For example, SAGA can be recruited to the promoters of ER stress target genes [23] and not to immediate early (IE) genes, where ATAC is found upon TPA induction [21]. Many proteins are involved in mediating and recovering from ER stress. The function of the GRP78 protein lies in the detection of mis-folded proteins that cause ER stress. GRP78 activates the PERK and ATF6 pathways, which in turn induce transcription of *CHOP* and *GRP78* via the ATF4 and ATF6 transcription factors. CHOP has further downstream functions in the ER stress response [31]. Interestingly, *in vitro* promoter binding studies show that ATF6α, an important transcription factor in the ER stress response, can bind and recruit both the SAGA and ATAC complexes to immobilized DNA templates [21]. When ER stress is induced *in vivo* by thapsigargin treatment, SAGA is recruited to the TSS of *GRP78* and *CHOP* and functional intact SAGA is required for proper transcription of these genes [32].

Here we examined the role of SGF29 in the recovery of human osteosarcoma cells from ER stress. We observed that the survival of cells after ER stress is reduced in SPT20 and SGF29 knockdown cells. This lower ER stress resistance correlates well with lower transcription induction of *GRP78* and *CHOP* and a lower H3K14 acetylation of their promoters. Interestingly also H3K4me3 levels of the *GRP78* and *CHOP* promoters are greatly decreased in SGF29 KD cells. The importance of H3K4me3 in the ER stress response is further stressed by the finding that knockdown of the H3K4me3-reader of TFIID, TAF3, results in similar, yet less pronounced, effects on gene induction and cell survival after ER stress. Reduced levels of H3K4me3 are concomitant with a reduced association of the SET1/MLL core subunit, ASH2L. We hypothesize that the concerted action of a number of transcriptional activators including TFIID, MLL and SAGA is required for maintaining stress response genes in a ‘poised’ chromatin state and facilitate their rapid, full activation upon stress induction.

## Materials and Methods

### Cell culture, knockdown, lentivirus infection and ER stress treatment

Human osteosarcoma cell line U2OS (#HTB-96), HeLaS3 (CCL-2.2) obtained at ATCC and HeLa FRT [33] cells were maintained as monolayers in normal glucose Dulbecco’s modified Eagle’s medium (DMEM, InVitrogen), containing 10% fetal bovine calf serum (FBS, Lonza) and 1% penicillin/streptavidin and L-glutamine (Lonza). pLKO-puro constructs (Sgf29 #1-TRCN0000141325, Sgf29 #2-TRCN0000144091, Taf3 #5.2 TRCN0000016608 and Taf3#5.3 TRCN0000016609) expressing shRNAs that target *SGF29* or *TAF3* mRNAs were obtained from Open Biosystems. As a control for the knockdown experiments, a non-targeting shRNA with the following sequence 5’- CCGGGCGAACAAGAAGAAGGACAAACTCGAGTTTGTCCTTCTTCTTGTTCGCTTTTT-3’ was used. Viral production was performed in Cos7 cells by transfection of 2 µg each of pRSV-rev, pMDLg/pRRE, pMD2.G, and pLKO-shRNA using Fugene 6 (Roche). Lentivirus containing medium was collected 48 h after transfection, filtered and concentrated by ultracentrifugation (2.5 hour, 76,000 g, 18°C). 2.5*10^6^ cells (U20S and HeLa FRT) were used for infection and puromycin selection was started two days later. U2OS were plated at low density for monoclonal outgrowth and colonies picked after 14 days of culturing. Stable GFP-tagged *SGF29*, *ASH2L* and *RBBP5* cell lines were created by cloning of the ORFs into pCDNA.5/FRT/TO (InVitrogen) and subsequent recombination into Hela FRT cells carrying the Tet repressor for inducible expression [23]. Endoplasmic reticulum (ER) stress was induced by the addition of 5 µg/µl tunicamycin (Sigma-Alldrich) to the growth medium for indicated times.

### Chromatin immunoprecipitation

Cells were cross-linked at 80-90% confluency using 1% paraformaldehyde in PBS for 10 min at room temperature. Reactions were quenched by addition of 125 mM glycine for 5 minutes on ice. After a cold PBS wash cells were scraped and collected by centrifugation (5 min, 400 g, 4ᵒC). Pelleted cells were resuspended in ChIP lysis buffer (1% SDS, 10 m1M EDTA, 50mM Tris-HCl pH 7.9, 1 mM DTT, 5 µM sodium butyrate (Merck) and complete protease inhibitors (Roche)) and disrupted by sonication (Bioruptor, Diagenode: seven cycles, 30 sec on/off, high setting) to produce an average DNA fragment size of ~ 400 bp. Samples were centrifuged (5 min, 200 g, 4ᵒC) and supernatant collected. For immunoprecipitation, chromatin was diluted in IP buffer (0.5% Triton X-100, 2 mM EDTA, 20 mM Tris-HCl pH 7.9, 150 mM NaCl, 1 mM DTT, 5 µM sodium butyrate and complete protease inhibitors (Roche)), 1-5 µg antibody was added and rotated overnight at 4ᵒC. Immunocomplexes were collected for 4 hrs at 4ᵒC on protein A/G PLUS-agarose beads (Santa-Cruz), after o/n blocking in 1.5% fish gelatin and washing. Subsequently beads were washed four times at 4ᵒC with wash buffer (0.25% NP-40, 0.05% SDS, 2 mM EDTA, 20 mM Tris-HCl pH 7.9, 250 mM NaCl, 5 µM sodium butyrate and complete protease inhibitors) and once with TE (10 mM Tris-HCl pH 6.8, 1 mM EDTA). Cross-links of protein-DNA were reversed by overnight incubation at 65ᵒC and eluted in 100 µl elution buffer (100 mM NaHCO_3_, 1% SDS). Samples were treated with 1 mg/ml proteinase K (Roche) and 1 mg/ml RNase A for 2 hours at 37ᵒC. DNA was purified using PCR purification kit (Qiagen) and amplified in a 25 µl reaction mixture (iQ SYBR green supermix (Biorad)) in a real-time PCR machine (CFX96, Biorad). Primer sequences are available upon request.

### Fluorescent-activated cell sorting (FACS) analysis

To measure apoptosis 2*10^5^ wildtype or knockdown U2OS cells were seeded in 6-well plates. After tunicamycin treatment, cells were washed twice with PBS and recovered overnight in normal DMEM. All cells were collected, centrifuged (10 min, 600 g, RT) and resuspended in PBS with 5 mg/ml propidium iodide and in some experiments Annexin V (InVitrogen). Cells were incubated 5 min on ice before analysis on a Becton Dickinson FACS Calibur.

### mRNA expression analysis

Total RNA was isolated using RNeasy kit (Qiagen) and cDNA was synthesized using the First-strand cDNA synthesis kit (Qiagen) both according to the manufacturers manual. Subsequently the cDNA was amplified in a 25 µl reaction mixture (iQ SYBR green supermix (Biorad)) in a real-time PCR machine (CFX96, Biorad). XBP1 mRNA was measured by RT-PCR. Samples were loaded on a 2% agarose gel and stained with ethidium bromide. Primer sequences are available upon request.

### SDS-PAGE, immunoblot analysis and antibodies

Whole cell lysates were analyzed by immunoblotting according to standard procedures. In short, cells were lysed and scraped in sample buffer and boiled at 95ᵒC for 5 min. Reactions were run on SDS-polyacrylamide gels and transferred to polyvinylidene difluoride membrane. Molecular mass markers were obtained from New England Biolabs. Antibodies used were anti-SGF29 [34], anti-tubulin (Calbiochem CP06), anti-H3 (Abcam Ab1791), anti-H3K4me3 (Diagenode pAB-003-050), anti-RBBP5 (Bethyl BL766), anti-ASH2L (gift from Winship Herr), anti-WDR5 (a gift from Winship Herr) and anti-GFP (a gift from Geert Kops). Additional antibodies used for ChIP are anti-H3K14ac [21], anti-H3K4me3 (Millipore 05-745R) and anti-H3K18ac (Abcam Ab1191).

## Results

### SAGA and SGF29 are involved in cell survival of U2OS cells after ER stress

Previous studies of SAGA and ER stress involved thapsigargin treatment of Hela cells, which is known to cause irreversible damage to cells [35]. Tunicamycin is a milder treatment to induce ER stress and in contrast to thapsigargin many human cell lines can recover from tunicamycin treatment using moderate doses [36]. We first tested the toxicity of tunicamycin on a human osteosarcoma cell line (U2OS). Following treatment of cells in increasing amounts, FACS analysis was performed to determine the survival rate of cells. The cells were treated for 4 or 8 hours with tunicamycin, or with DMSO as a control. Non-fixed cells were then treated with propidium iodide (PI), which stains the DNA of cells with disrupted membranes such as necrotic or apoptotic cells. Increasing the amount of tunicamycin resulted in a mild increase in PI positive cells after 8 hours of treatment (Figure 1A). This indicates that the amount of apoptotic cells is negligible at all tested tunicamycin concentrations. We also investigated cell recovery after tunicamycin treatment by monitoring restoration of unspliced XBP1 mRNA. XBP1 splicing by IREp is an early step in the ER stress response, leading to increased amounts of the (smaller) spliced variant [37]. Upon recovery from ER stress the amount of the unspliced variant should be restored. U2OS WT cells were treated for the indicated times with 5 µ/ul tunicamycin and XBP1 mRNA was measured by RT-PCR (Figure 1B). The unspliced XBP1 isoform starts being restored after 8 hours of treatment and full restoration is observed after 24 hours of tunicamycin treatment. These results indicate that U2OS cells are capable of responding to this dose of tunicamycin.

**Figure 1:** SPT20 and SGF29 are required for cell survival after ER stress in U2OS cells. U2OS cells were transduced with lentiviruses targeting *SPT20* or *SGF29* (two different shRNAs) or a non-target control shRNA. **A**. Different amounts of tunicamycin were tested for toxicity in U2OS WT cells. Schematic representation of FACS results of propidium (PI) positive cells. **B**. Recovery of unspliced XPB1 mRNA in U2OS wt cells after tunicamycin treatment (5ug/ul) for indicated times. Amount of XPB1 mRNA is measured by RT-PCR. **C**. and **E**. Analysis of mRNA expression levels of *SPT20* and *SGF29* by quantitative RT-PCR, corrected for *β-ACTIN*. Standard deviations represent technical triplicates. **D**. and **F**. Schematic representation of FACS results, increase in PI positive cells upon SPT20 knockdown (KD) and increase of PI- and annexin V-positive cells upon SGF29 KD. Samples were measured after 8 hours treatment with tunicamycin or DMSO followed by an o/n recovery. Standard deviations represent technical duplicates. Similar results were observed in two independent experiments.

SGF29 is responsible for binding SAGA to the H3K4me3 modification on ER stress target gene promoters, thus we decided to investigate the involvement of SGF29 in cell survival and gene activation after ER stress induced by tunicamycin. To first examine ER stress dependence on SAGA in this cell system, SPT20 kd cells were created by lentiviral transduction of two independent short hairpin (sh) RNAs targeting *SPT20* or as a control, a non-targeting hairpin (Figure 1C). A FACS based assay was used to determine the survival rate of cells from tunicamycin. The cells were treated for 8 hours with tunicamycin, or with the DMSO carrier only, and allowed to recover overnight. Non-fixed cells were treated with PI, FACS analysis reveals a higher percentage PI-positive cells in SPT20 knockdown (kd) cells (24% and 16%) than the control kd cells (5%) after tunicamycin treatment and recovery from ER stress (Figure 1D). This observation correlates well with the reduced ER stress gene induction in HeLa cells [38] and indicates that SPT20 (and most likely the SAGA complex) plays a general role in the ER stress response pathway of human cells.

Having established the U2OS system to study ER stress induction by tunicamycin, we focused on the SGF29 protein, which is a subunit of both the SAGA and ATAC complex. An important feature of both SAGA and ATAC is the ability to bind to chromatin and more specifically, to the H3K4me3 modification. This interaction is mediated by SGF29 [25,28]. To investigate a potential role for Sgf29 in the ER stress response, a U2OS cell line with a stable knockdown of SGF29 was created (Figure 1E). SGF29 or control KD cells were assayed for survival from ER stress by FACS analysis for PI- and annexin V-staining after tunicamycin treatment. As was observed in SPT20 kd cells, SGF29 kd cells showed a higher staining both for PI and for annexin V (25% and 37% vs. 6%) detecting apoptotic cells (Figure 1F), suggesting not only SAGA activity, but also specific recruitment to H3K4me3 is required for its role in ER stress survival.

### SGF29 protein is required for induction and H3 acetylation of ER stress genes

Given the fact that reduction of SGF29 and SAGA yielded similar effects on ER stress survival and SPT20 binds to the promoters of ER stress target genes *GRP78* and *CHOP* [23], we further investigated the role of SGF29 in this process. ER stress was induced by tunicamycin and mRNA levels of *GRP78* and *CHOP* were determined. SGF29 KD resulted in lower gene activation upon ER stress (Figure 2A).

**Figure 2:** The SGF29 protein is recruited to ER stress target genes and required for acetylation and subsequent transcription induction. A. Analysis of mRNA expression levels of *GRP78* and *CHOP* by quantitative RT-PCR. Levels were normalized to β-ACTIN and are presented as change compared to a control DMSO-treated sample. Samples were analyzed 4 and 8 h after tunicamycin treatment. B. Immunoblot analysis for doxycycline-inducible GFP-SGF29 and endogenous SGF29. C. Localization of the primer pairs used for ChIP. D. ChIP analysis of GFP-SGF29. On the x-axis are indicated amplicons for the *GRP78* and *CHOP* genes or a non-coding control region. Cells were not treated (T0, black histograms) or treated for 4 h with tunicamycin (t=4, white bars). Standard deviations represent technical triplicates and similar results were observed in at least three independent experiments. E. H3K14ac ChIP (percentage of input relative to H3 ChIP) at the transcription start site of ER stress target genes and a non-coding control region for 0 and 4 hours treatment with tunicamycin. Standard deviations represent technical triplicates and similar results were observed in at least two independent experiments.

To facilitate chromatin immunoprecipitation (ChIP) using a GFP-antibody, a doxycycline-inducible cell system for GFP-SGF29 expression was created (Figure 2B). Multiple primer pairs were designed to detect GFP-SGF29 binding to ER stress target genes (Figure 2C). After GFP-SGF29 expression was established by the addition of doxycycline, ER stress was induced by a 4-hour tunicamycin treatment. GFP-SGF29 binding was detected close to the transcription start sites (TSS) of *GRP78* and *CHOP* both prior to and after tunicamycin treatment (Figure 2D). GFP-SGF29 was not detected with primer pairs distal to the TSS, nor to a non-coding control region. Upon tunicamycin treatment (t=4), GFP-SGF29 binding to the TSS is increased about two-fold (Figure 2D). Previously, recruitment of the SAGA subunits SPT20, SPT3 and ATXN7L3 was reported, as was a functional requirement of SPT20 for transcriptional induction. Together, these and previous results suggest that SGF29 and the SAGA complex binds to these genomic loci.

SGF29 could be important for the recruitment of SAGA to the ER stress target genes and subsequent induction. In this scenario, SGF29 depletion may result in lower levels of H3 acetylation on the *GRP78* and *CHOP* promoters. Indeed, we observed reduced induction of H3K14ac in the absence of SGF29 (Figure 2E), which is in agreement with data obtained in yeast [28]. Together these results reveal a central role for SGF29 in the ER stress survival, ER stress target gene acetylation and induction.

### H3K4me3 on ER stress target genes is SGF29-dependent and TAF3 is also required for proper gene induction and cell survival

The results presented thus far indicate that SGF29 depletion results in a reduced binding of SAGA to ER stress genes. Since SGF29 binds to H3K4me3 and H3K4me3 is related to active transcription, we determined the levels of H3K4me3 during ER-stress induction (Figure 3A). To our surprise, the levels of H3K4me3 in SGF29 KD cells are reduced at the *GRP78* and *CHOP* promoters (Figure 3A) independent of ER stress, while global levels of H3K4me3 are not affected (Figure 3B). In contrast to H3K14ac, H3K4me3 is already present at the *GRP78* and *CHOP* promoters before (t=0) tunicamycin induction. These results indicate that the H3K4me3 mark is established independent of ER stress and prior to transcriptional induction. Recently it was shown that TAF3, the TFIID subunit that binds to H3K4me3 [15] regulates specific sets of target genes upon DNA-damage stress [18]. [18]. We therefore hypothesized that ER stress target genes could display a similar dependence on TAF3 and H3K4me3. To test a potential requirement for TAF3 in ER stress, stable TAF3 KD cell lines were created through transduction of two independent shRNA constructs targeting *TAF3* (Figure 3C). Indeed, *GRP78* and *CHOP* induction after tunicamycin treatment was lower after TAF3 knockdown (Figure 3D). FACS analysis of PI stained cells showed that TAF3 knockdown increased the percentage of apoptotic cells after tunicamycin treatment compared to the control cells (Figure 3E). Interestingly, however, H3K4me3 levels are not affected in TAF3 KD cells and do not significantly change upon ER stress induction (Figure 3F). These findings suggest that the TAF3-H3K4me3 interaction is not essential for maintaining ER stress response genes in a ‘poised’ state, but rather has a role in the full transcriptional activation upon ER stress and subsequent cell survival.

**Figure 3:** SGF29 regulates H3K4me3 levels on ER stress target genes and TAF3 is also involved in the ER stress response. ChIP of H3K4me3 and U2OS cells transduced with lentiviruses carrying *TAF3* or non-target control shRNAs. **A**. H3K4me3 ChIP (percentage of input relative to H3 ChIP) at the transcription start site of ER stress target genes and a non-coding control region for 0 and 4 hours treatment with tunicamycin. Standard deviations represent technical triplicates and similar results were observed in at least three independent experiments. **B**. Immunoblot analysis of proteins from SGF29 KD cells for global levels of H3K4me3. **C**. Analysis of mRNA expression of *TAF3* by quantitative RT-PCR, corrected for *β-ACTIN* and standard deviations represent technical triplicates. **D**. Analysis of mRNA expression levels of *GRP78* and *CHOP* by quantitative RT-PCR. Levels were normalized to β-ACTIN and are presented as change compared to a control DMSO-treated sample. Samples were analyzed 4 and 8 h after tunicamycin treatment. **E**. Schematic representation of FACS results, increase in propidium (PI) positive cells in *TAF3* kd cells after tunicamycin treatment. Samples were measured after 8 hours treatment with tunicamycin or DMSO and o/n recovery. Standard deviations represent technical duplicates. Similar results were observed in two independent experiments. **F**. H3K4me3 ChIP (percentage of input relative to H3 ChIP) at the transcription start site of ER stress target genes and a non-coding control region for 0 and 4 hours treatment with tunicamycin. Standard deviations represent technical triplicates and similar results were observed in at least two independent experiments.

### SGF29 and the recruitment of H3K4 methyltransferase complexes

The ChIP results indicate involvement of SGF29 in maintenance of H3K4me3 at ER stress target genes. The reduction in H3K4me3 could be due to either reduced H3K4 methylation or increased turnover. To explore this further we examined involvement of the SET1/MLL methyltransferase complexes, responsible for the bulk H3K4me3 in mammalian cells [39], at the ER stress target genes. Global levels of ASH2L, RBBP5 and WDR5, core subunits of these methyltransferase complexes [18] showed no decrease in SGF29 KD cells (Figure 4A). Next, we employed the doxycycline-inducible system to create GFP-ASH2L or GFP-RBBP5 cell lines for ChIP analysis (Figure 4B). ChIP analysis indicated that ASH2L and RBBP5 associate to the TSS of *GRP78* and *CHOP* (Figure 4C) at the same location as SGF29 (Figure 2D). To test the effect of SGF29 KD on the localization of MLL complex on ER stress genes, we knocked down SGF29 in GFP-ASH2L cells (Figure 4D). SGF29 KD does not affect the levels of doxycycline-induced GFP-ASH2L expression (Figure 4E). Strikingly, we observed a significant decrease of GFP-ASH2L at the *GRP78* and *CHOP* promoter in the absence of SGF29 (Figure 4F). These results suggest involvement of SGF29 and SET1/MLL complexes for maintenance of H3K4me3 levels prior to ER stress, thereby prompting rapid transcriptional induction in an ER stress situation

**Figure 4:** ASH2L and RBBP5 associate to *GRP78* and *CHOP* promoters and ASH2L binding is SGF29 dependent. ChIP of ASH2L and RBBP5 at the transcription start site of the *GRP78* and *CHOP* genes. **A**. Immunoblot analysis of proteins from SGF29 KD cells for global levels of SET1/MLL subunits ASH2L, RBBP5 and WDR5. **B**. Immunoblot analysis of protein levels of inducible GFP-ASH2L and GFP-RBBP5 and endogenous RBBP5. **C**. ChIP analysis of GFP-ASH2L and GFP-RBBP5. Standard deviations represent technical triplicates and similar results were observed in at least three independent experiments. **D**. Analysis of mRNA expression of *SGF29* by qPCR, corrected for *β-ACTIN* and standard deviations represent technical triplicates. **E**. Immunoblot analysis of GFP-ASH2L protein levels in GFP-ASH2L cell line infected with non target (lane 1 and 2) and *SGF29* hairpin (lane 3 and 4). **F**. ChIP analysis of GFP-ASH2L in control and SGF29 KD lines. Standard deviations represent technical triplicates and similar results were observed in at least three independent experiments.

## Discussion

In this study we have uncovered an important role for SGF29, subunit of HAT coactivator complexes SAGA and ATAC, in the human ER stress response. We find that SAGA is important for cell survival after ER stress in multiple cell systems, since SPT20 knockdown leads to lower survival rates (Figure 1A). SGF29 KD cells also display a decreased resistance to ER stress (Figure 1D), while SGF29 might be central in recruiting a HAT complex to the H3K4me3 on the stress gene promoters. It is important to mention that SGF29 is part of both SAGA and ATAC. The composition of the HAT module of ATAC is highly similar to the SAGA HAT module and the main difference is that ADA2B is replaced by ADA2A [5,40,41]. SAGA seems to have a preference for promoters, while ATAC is more found on enhancers [30]. Interestingly, ATAC subunits were not identified to bind to H3K4me3 peptides in human cell extracts [42]. However, ATAC was found to bind H3K4me3 peptides in different mouse tissue extracts [25] and *in vitro* ATF6 mediates recruitment of both SAGA and ATAC to the immobilized *GRP78* promoter [43]. Based on these studies it is possible that (part of) the effects we observe in SGF29 KD cells are not only dependent on the recruitment of SAGA, but may also involve the ATAC complex. Future experiments including specific subunit analysis of both SAGA and ATAC at multiple ER stress genes will resolve this issue. It has been shown previously that SPT20 recruitment to ER stress gene promoters is clearly linked to the transcriptional induction of these genes [31]. Their impaired induction upon SPT20 or SGF29 knockdown would affect recovery from ER stress and decrease cell survival. Since SGF29 is responsible for binding of SAGA to H3K4me3 [23], the fact that SGF29 loss results in similar effects as SPT20 knockdown (our results and [25,28] suggests that SAGA binding to H3K4me3 via its SGF29 subunit has a central role in the function of HAT complexes in the ER stress response. The effects observed on the H3K14ac of the *GRP78* and *CHOP* promoters in SGF29 KD cells underscores this role.

SGF29 forms a mechanistic basis for crosstalk between histone modifications like H3K4 methylation and H3 acetylation and how this is linked to active transcription of ER stress genes. It is interesting to note that the activation of DNA damage genes requires a different HAT complex, but employs a similar mechanism. For these genes the PHD finger-containing ING4 subunit of the HBO1 HAT complex links H3K4me3 and H3 acetylation with transcriptional activation of these genes [44]. H3K4me3 is already present before ER stress treatment on the *GRP78* and *CHOP* promoters and its levels do not increase during transcriptional induction in human U2OS osteosarcoma cells (Figure 4A). These results mirror previous findings of a constitutive H3K4 methylation of the *CHOP* locus in human HepG2 hepatoma cells [45]. Similar to the ER stress gene promoters the DNA-damage inducible *SMC4* promoter also carries the H3K4me3 mark prior to activation [44]. This implies that binding of SAGA to a promoter is not solely dependent on SGF29. This is not surprising since SAGA was previously shown to be recruited to promoters by transcription factors such as ATF6 [31]. Furthermore, the TRRAP subunit of SAGA can directly interact with c-myc and other activator proteins [46,47].

The role of SGF29 in human cells is more complicated than simply anchoring SAGA to H3K4me3-modified nucleosomes as was proposed for yeast SGF29 [28]. Depletion of human SGF29 also results in a reduction of H3K4me3 from ER stress gene promoters. This decrease of H3K4me3 was unexpected since SGF29 is mainly regarded as a downstream effector for this mark. What could be the mechanistic basis for this? Our ChIP analyses indicate involvement of the SET1/MLL methyltransferase complexes as ASH2L and RBBP5 associate to the *GRP78* and *CHOP* promoters also prior to ER stress. The expression of ASH2L and RBBP5 is not reduced in SGF29 KD cells but the association of these SET1/MLL core subunits to the *GRP78* and *CHOP* promoters is affected. Future experiments should be aimed at identifying the specific SET1/MLL complexes involved in ER stress gene transcription and how SGF29 and SAGA is involved in their recruitment. In summary, our results reveal a sophisticated and fine-tuned interplay between distinct chromatin modifying enzymes and the basal transcription machinery, which is required for the prompt activation of target genes in response to stress
